# PDP1 Promotes Cell Malignant Behavior and Is Associated with Worse Clinical Features in Ovarian Cancer Patients: Evidence from Bioinformatics and In Vitro Level

**DOI:** 10.1155/2022/7397250

**Published:** 2022-10-14

**Authors:** Yan Song, Juan Zhang, Lei Zhang, Suxia Zhang, Chengcheng Shen

**Affiliations:** ^1^Jinan Maternity and Child Care Hospital Affiliated to Shandong First Medical University, Jinan, Shandong, China; ^2^Liaocheng People's Hospital, Liaocheng, Shandong, China

## Abstract

PDP1 has been reported in multiple diseases. However, it has not been fully explored in ovarian cancer (OC). The public data was downloaded from The Cancer Genome Atlas (TCGA) and Gene Expression Omnibus (GEO) databases. Differentially expressed gene analysis was conducted out using the limma package. Prognosis analysis was performed using the survival package. Gene Set Enrichment Analysis (GSEA) was performed using the fgsea package. Immune infiltration analysis was performed based on the CIBERSORT algorithm. CCK8 assay was used to evaluate the cell proliferation ability of cancer cells. Transwell assay was used for the invasion and migration ability. Our result showed that PDP1 was overexpressed in OC tissue in RNA and protein level based on multiple databases (TCGA, GSE18520, GSE27651, and GSE54388). At the same time, we found PDP1 was correlated with poor prognosis and worse clinical parameters. In vitro experiment showed that PDP1 could significantly promote proliferation, invasion, and migration ability of OC cells. GSEA analysis showed that in the OC patients with high PDP1 expression, the pathway of IL6/JAK/STAT3 signaling, interferon-alpha response, apoptosis, adipogenesis, KRAS signaling, and IL2/STAT5 signaling was activated, which might be responsible for its oncogenic effect in OC. Immune infiltration analysis indicated that PDP1 was positively correlated with activated myeloid dendritic cells, resting CD4 memory T cells, neutrophil, and M1 and M2 macrophages, yet negatively correlated with M0 macrophages, plasma B cells, *γδ*T cells, and activated CD4 memory T cells. Drug sensitivity analysis showed a negative correlation between PDP1 expression and the IC50 of bleomycin and gemcitabine, yet a positive correlation of cisplatin, indicating that the OC patients with high PDP1 expression might be more sensitive to bleomycin and gemcitabine and more resistant to cisplatin. PDP1 could facilitate OC progression and is associated with patient prognosis and chemosensitivity, making it an underlying biomarker of OC.

## 1. Introduction

Ovarian cancer (OC) is a common malignancy with a rising trend of morbidity in females, making it a major health concern worldwide [1]. As a heterogeneous disease, OC has characteristics of high incidence and high mortality rate. During the past decades, the five-year survival rate of OC remained below 50%, and no significant improvement was observed along with the advancement of medical conditions [2]. Meanwhile, due to the insidious symptoms, the early deletion of OC is difficult to complete, and a significant number of patients presented advanced stage at diagnosis [3]. Therefore, it is meaningful to identify novel and effective biomarkers for OV early detection and treatment.

Pyruvate dehydrogenase phosphatase catalytic subunit 1 (PDP1) encodes the protein that is one of the three components (E1, E2, and E3) of the large pyruvate dehydrogenase complex [4]. PDP1 plays an important role in protein phosphorylation [4, 5]. The biological role of PDP1 was also observed in multiple diseases. Shi and colleagues demonstrated that the PDP1-PDH-histone acetylation retrograde signaling activated by mitochondrial dysfunction could significantly increase the radioresistance in colorectal cancer [6]. Feng and colleagues found that miR-18a-3p could improve cartilage matrix remodeling and inhibit inflammation in osteoarthritis by suppressing PDP1 [7]. In pancreatic cancer, Li and colleagues found that PDP1 promotes pancreatic cancer proliferation and invasion through regulating the MAPK/mTOR signaling pathway [8]. Shan and colleagues revealed that phosphorylation of the Tyr-94 site could hamper PDP1 expression and facilitate the growth of leukemia cells [9]. A comprehensive review conducted by Jeoung concluded that pyruvate dehydrogenase kinases (PDKs) and pyruvate dehydrogenase phosphatases (PDPs) have unique tissue-specific expression, kinetic properties, and sensitivity to regulatory molecules, which might be therapeutic targets for diabetes and cancers [10]. Chen and colleagues PDP1 was associated with the prognosis of breast cancer patients and their immune microenvironment [11]. Moreover, Chen and colleagues found that PDP1 was overexpressed in prostate cancer and could sustain prostate tumorigenesis by controlling lipid biosynthesis [12]. However, the underlying role of PDP1 in OC has been thoroughly studied.

Our study systematically investigated the role of PDP1 in OC. PDP1 was upregulated in OC tissue and cell lines, which was associated with worse clinical features and poor prognosis. In vitro experiment showed that PDP1 could promote proliferation, invasion, and migration of OC cells. GSEA and immune infiltration analysis were performed to explore the underlying pathway and immune microenvironment difference between low and high PDP1 patients. Moreover, we found that PDP1 could affect the sensitivity of chemotherapy, making it a potential therapeutic target of OC patients.

## 2. Results

### 2.1. Identification of the Common Differentially Expressed Genes (DEGs) between OC and Normal Tissue

The flow chart of the whole study was shown in Figure 1. Firstly, we performed DEG analysis between the OC and normal ovarian tissue based on the data of GSE18520, GSE27651, and GSE54388. GSE18520 identified 1009 upregulated and 1554 downregulated genes (Figure 2(a)); GSE27651 identified 1966 upregulated and 2553 downregulated genes (Figure 2(b)); GSE54388 identified 625 upregulated and 743 downregulated genes (Figure 2(c)). Meanwhile, we performed univariate Cox regression analysis to identify the prognosis-related genes. Commonly upregulated genes intersect the genes with HR > 1 and finally identified five genes, KLHL14, SLC4A11, S100A2, PDP1, and TMC4 (Figure 2(d)). Commonly downregulated genes intersect the genes with HR < 1 and finally identified six genes, ITLN1, HSD17B2, FGF13, ME1, TNFSF13B, and AADAC (Figure 2(e)).

### 2.2. Exploration of the Expression Pattern of PDP1 in OC

Pan-cancer analysis based on TCGA and GTEx data showed that PDP1 has an aberrant expression analysis in most cancers, including OC (Figure 3(a)). Also, we observed a higher expression level of PDP1 in OC tumor tissue in multiple cohorts, consisting of TCGA + GTEx, GSE18520, GSE27651, and GSE54388 (Figures 3(b)–3(e)). Further, we evaluate the protein level of PDP1 through the IHC images obtained from the HPA database. The result indicated that PDP1 also had a higher protein level in OC tumor tissue compared with the normal tissue (Figures 3(f) and 3(g)).

### 2.3. PDP1 Might Be Prognosis and Clinical Biomarker of OC

Next, we evaluate the PDP1 expression in OC patients with diverse clinical features. We found that the OC patients with lymphatic invasion, venous invasion, and worse clinical-stage tend to have a higher PDP1 expression (Figures 4(a)–4(c)). Although the statistical was not significant, considering the small sample bias, we still considered that the PDP1 was associated with worse clinical features. Moreover, we found that the OC patients with higher PDP1 level have a poor OS, DSS, and PFI (Figures 4(d)–4(f); overall survival, HR = 1.32, *P* = 0.039; disease-specific survival, HR = 1.27, *P* = 0.1; progress-free interval, HR = 1.24, *P* = 0.071). Furthermore, a receiver-operating characteristic (ROC) curve was used for quantifying the predictive ability of patient prognosis. The result showed that PDP1 might have a satisfactory prognosis prediction ability for the OS, DSS, and PFI of OC patients (Figure 4(g), OS, 1-year AUC: 0.580, 3-year AUC: 0.725, 5-year AUC: 0.700; Figure 4(h), DSS, 1-year AUC: 0.558, 3-year AUC: 0.723, 5-year AUC: 0.697; Figure 4(i), 1-year AUC: 0.627, 3-year AUC: 0.760, 5-year AUC: 0.787). Univariate and multivariate analysis indicated that PDP1 is a risk factor independent of other clinical features (Figures 4(j) and 4(k)).

### 2.4. PDP1 Promotes Proliferation, Invasion, and Migration of OC Cells

To explore the underlying biological role of PDP1 in OC, we performed in vitro experiments to assess the influence of PDP1 on OC cell malignant behaviors. The qRT-PCR result showed a higher PDP1 level in OC cell lines than the normal IOSE80 cells (Figure 5(a)). An effective knockdown of PDP1 was also observed in selected A2780 and SKOV3 cell lines (Figures 5(b) and 5(c)). CCK8 assay showed that the inhibition of PDP1 could significantly suppress the proliferation ability of OC cells (Figures 5(d) and 5(e)). Moreover, the Transwell assay showed that the knockdown the PDP1 could remarkably inhibit the invasion and migration of OV cells (Figure 5(f)).

### 2.5. PDP1 Activated Multiple Oncogenic Signaling in OC

GSEA analysis was performed to explore the potential biological difference between low and high PDP1 OC patients. The result showed that in the OC patients with high PDP1 expression, the pathway of IL6/JAK/STAT3 signaling, interferon-alpha response, apoptosis, adipogenesis, KRAS signaling, and IL2/STAT5 signaling was activated, which might be responsible for its oncogenic effect in OC (Figure 6(a)). Gene Ontology (GO) analysis in the patients with high PDP1 expression, the terms of cellular response to prostaglandin E stimulus, negative regulation of activated T cell proliferation, positive regulation of macrophage differentiation, regulation of extracellular matrix assembly, and regulation of membrane invagination were significantly enriched (Figure 6(b)). Kyoto Encyclopedia of Genes and Genomes (KEGG) analysis showed that in the patients with high PDP1 expression, terms of glycosphingolipid biosynthesis lacto and neolacto series, allograft rejection, graft versus host disease, and colorectal cancer were mainly enriched in (Figure 6(c)).

### 2.6. PDP1 Acted as an Immune-Related Gene and Was Associated with Chemosensitivity

The tumor immune microenvironment plays an important role in tumorigenesis and tumor development. Therefore, we explored the effect of PDP1 on the tumor immune microenvironment. CIBERSORT algorithm was used for immune cell quantification. The result showed that PDP1 was positively correlated with activated myeloid dendritic cells, resting CD4 memory T cells, neutrophil, and M1 and M2 macrophages, yet negatively correlated with M0 macrophages, plasma B cells, *γδ*T cells, and activated CD4 memory T cells (Figure 7(a)). Bleomycin, gemcitabine, cisplatin, and paclitaxel were the frequent chemotherapy regimen of OC. We further investigated the influence of PDP1 on the chemosensitivity of these drugs based on the GDSC database. Drug sensitivity analysis showed a negative correlation between PDP1 expression and the IC50 of bleomycin and gemcitabine, indicating that the OC patients with high PDP1 expression might be more sensitive to bleomycin and gemcitabine (Figures 7(b) and 7(c); bleomycin: *R* = −0.23, *P* < 0.001; gemcitabine: *R* = −0.10, *P* = 0.048). In contrast, cisplatin showed opposite results (Figure 7(d); cisplatin: *R* = 0.35, *P* < 0.001). Meanwhile, no significant effect was observed in paclitaxel (Figure 7(e)).

## 3. Discussion

As one of the most threatening malignant tumors in females, OC still has high incidence and mortality despite the advancement of medicine [13]. For advanced OC, the therapeutic effects are not satisfactory currently. Targeted therapy is a promising therapeutic strategy for progressive OC. Therefore, it is necessary to identify the novel target with potential for clinical translation.

To the best of our knowledge, this study was the first study comprehensively exploring the role of PDP1 in OC. Here, we found that PDP1 was overexpressed in OC tissue and cells, which was associated with more progressive clinical features and poor prognosis. Moreover, the knockdown of PDP1 could significantly suppress the cell malignant behavior of OC cells. Multiple oncogenic pathways were abnormally activated in high PDP1 patients. Meanwhile, PDP1 was remarkably correlated with several immune cells and might affect the chemosensitivity of OC patients.

PDP1 is a key regulator of pyruvate dehydrogenases complex (PDC) and can positively regulate the catalytic activity of PDC through mediating the dephosphorylation from the serine sites on E1*α* of the complex [14]. After being activated by PDP1, PDC could catalyze the oxidative decarboxylation of pyruvate to acetyl-CoA, which is a major energy-producing substrate [10]. Aberrant PDP1 level might lead to cell energy metabolism disorders, affecting cell malignant biological behaviors. The cancer-promoting effect of PDP1 on cancer cells was observed in multiple cancers, including colon cancer, prostate cancer, and nonsolid tumor [6, 9, 12]. Our study fills the gap of PDP1 in OC, and the result showed that PDP1 could promote OC progression, making it an underlying therapeutic target.

GSEA result showed that the pathway of IL6/JAK/STAT3 signaling, interferon-alpha response, apoptosis, adipogenesis, KRAS signaling, and IL2/STAT5 signaling was activated in high PDP1 patients. IL6/JAK/STAT3 signaling was reported to facilitate cancer progression in multiple cancer. Ni and colleagues found that miR-515-5p could suppress the migration and invasion of liver cancer cells through targeting IL6/JAK/STAT3 pathway [15]. In gastric cancer, Zhao and colleagues indicated that IL6 could promote proliferation, invasion, and lymphangiogenesis by regulating the JAK/STAT3/VEGF-C signaling [16]. Moreover, Salimian and colleagues found that the omental adipose stromal cells could increase the nitric oxide level in OC cells, leading to the decrease of mitochondrial and enhanced cell malignant behavior [17]. KRAS mutation is the most frequently mutated RAS, which could activate downstream signaling and promote tumorigenesis [18]. Rahman and colleagues revealed that the gene amplification of KRAS and MAPK1 was essential for type II ovarian carcinomas' growth [19]. Wang and colleagues indicated that the MGP protein could directly bind to the p-STAT5 in the nucleus and activate JAK2/STAT5 signaling in gastric cancer, further facilitating tumor progression [20]. Our result showed that the cancer-promoting effect of PDP1 in OC might be dependent on these oncogenetic pathways.

Recently, increased attention has been paid to the effect of the tumor microenvironment on cancer cells [21]. The immune infiltration result showed that PDP1 was positively correlated with activated myeloid dendritic cells, resting CD4 memory T cells, neutrophil, and M1 and M2 macrophages, yet negatively correlated with M0 macrophages, plasma B cells, *γδ*T cells, and activated CD4 memory T cells. Neutrophils are increasingly acknowledged to contribute to tumor development [22]. Xiao and colleagues found that the CTSC could promote lung metastasis of breast cancer through mediating recruitment of neutrophils and formation of neutrophil extracellular traps based on the CTSC/PR3/IL-1*β* axis [23]. In OC, Lee and colleagues revealed that neutrophils could facilitate OC premetastatic niche formation in the omentum, therefore resulting in an environment favorable for cancer cells to implant [24]. Meanwhile, Zeng and colleagues found that M2-like tumor-associated macrophages-secreted EGF could facilitate epithelial OC metastasis by activating EGFR-ERK signaling and suppressing lncRNA LIMT expression [25]. Therefore, the underlying interaction between PDP1 and these immune cells might be partly responsible for the cancer-promoting effect of PDP1 in OC. Drug sensitivity analysis showed the OC patients with high PDP1 expression might be more sensitive to bleomycin and gemcitabine, which increase its potential for clinical application.

Although our study was based on reliable analysis, some limitations should be noticed. Firstly, the populations enrolled in our analysis were mainly the Western world individuals, and the race bias was inevitable. Secondly, the clinical information of OC patients in TCGA was incomplete, only including the grade and clinical stage. If the clinical information was more complete, the conclusion of our study would be more credible.

## 4. Conclusions

Based on the high-quality bioinformatics analysis and in vitro experiments, we found that PDP1 was overexpressed in OC tissue and cell lines. Moreover, PDP1 could significantly promote cancer cell proliferation, invasion, and migration. GSEA analysis showed that PDP1 could activate several oncogenic pathways, like IL6/JAK/STAT3 signaling and KRAS signaling. Immune infiltration analysis showed that PDP1 was positively correlated with activated myeloid dendritic cells, resting CD4 memory T cells, neutrophil, and M1 and M2 macrophages, yet negatively correlated with M0 macrophages, plasma B cells, *γδ*T cells, and activated CD4 memory T cells. Also, PDP1 was associated with the chemosensitivity of bleomycin, gemcitabine, and cisplatin.

## 5. Methods

### 5.1. Public Data Acquisition and Processing

All the data used for analysis were downloaded from The Cancer Genome Atlas (TCGA) and Gene Expression Omnibus (GEO) databases. For the TCGA database, the transcriptomic profiling (https://portal.gdc.cancer.gov/, TCGA-OV, date category: transcriptome profiling, data type: gene expression quantification, workflow type: FPKM) and clinical information (TCGA-OV, date category: clinical, data format: bcr xml) of OC patients were obtained from the TCGA-GDC server. The FPKM file was then converted into TPM form for further analysis. Data was collated and preprocessed using the R software. For the GEO database, the datasets GSE18520 (platform: GPL570), GSE27651 (platform: GPL570), and GSE54388 (platform: GPL570) were downloaded for analysis. The patients with complete gene expression profile and clinical information were included in our analysis. Limma package was used for differential expressed gene (DEG) analysis with the threshold of ∣logFC > 1∣ and *P* value < 0.05 [26]. The immunohistochemistry (IHC) pictures of PDP1 in OC tumor and normal tissue was obtained from The Human Protein Atlas (HPA) database. Survival analysis of PDP1 was performed using the survival package in R software. Gene set enrichment analysis was performed to explore the biological pathway difference between low and high PDP1 OC patients and the reference file was Hallmark, c2.cp.kegg.v7.5.1.symbols, and c5.go.v7.5.1.symbols pathway set. Immune infiltration analysis was performed using the CIBERSORT algorithm [27]. Drug sensitivity analysis was conducted out based on the Genomics of Drug Sensitivity in Cancer (GDSC) database.

### 5.2. Cell Culture and Transfection

The human normal ovarian epithelial cell line (IOSE80) and human epithelial ovarian cancer cell lines (CaOV-3, HO-8910, SKOV3, and A2780) were laboratory stocks. Cells were cultured in the conventional incubator atmosphere containing 5% CO2 at 37°C and routinely passaged three times weekly. Cell transfection was performed using the Lipofectamine 2000 according to standard protocol. PDP1 knockdown and control plasmids were purchased from Shanghai Jikai Gene Chemical Co., Ltd., whose target sequence were as follows: shRNA1: 5′-GCCTGTTTAATGGATATGTTT-3′; shRNA2: 5′-CTGTTAAAGTTTGTCAATTAA-3′; shRNA3: 5′-GACGATAAAGTGTTTTTAGTA-3′.

### 5.3. Quantitative Real-Time PCR (qRT-PCR)

A TRIzol RNA extraction kit (TaKaRa) was used to extract the total RNA following the protocol. Total RNA was then reverse-transcribed to cDNA. qRT-PCR was performed based on the SyBr Green system. The primer used was as follows: PDP1, forward, 5′-GTCCTTCCCATTCTGCAACC-3′; reverse, 5′-GAAACAGAGGAGGACCAAACA-3′, GAPDH, forward, 5′-GCAAATTCCATGGCACCGT-3′; reverse, 5′-TCGCCCCACTTGATTTTGG-3′.

### 5.4. CCK8 Assay

CCK8 assay was performed using a CCK8 Kit (Dojindo, Shanghai, China) according to the protocol. Cells were plated in a 96-well plate and added with a CCK8 solution. After that, cells were incubated for 1 h at 37°C, and then, the absorbance was detected at A450 nm for 0 h, 24 h, 48 h, and 72 h.

### 5.5. Transwell Assay

Transwell assay was performed using the Transwell chamber (8 *μ*m pore size, Corning). The Transwell chamber was added into the 24-well plates and divided into the compartment into the upper and lower chambers. The upper chamber was added with cells with 500 *μ*l in serum-free medium, and the lower chamber was added with 600 *μ*l complete media. After that for 24 h, cells were fixed with paraformaldehyde and stained with crystal violet.

### 5.6. Statistical Analysis

Statistical analysis was performed using the R software and GraphPad Prism 8. *P* value less than 0.05 was regarded as statistically significant. Student's *T* test was used for variables with normal distribution, and Wilcoxon test was used for variables with nonnormal distribution. All the experiments were repeated at least three times.

## Figures and Tables

**Figure 1:** The flow chart of the whole study.

**Figure 2:** Identification of differentially expressed genes between ovarian cancer and normal tissue. Notes: (a) differentially expressed gene analysis was performed under the threshold of ∣logFC > 1∣ and *P* value < 0.05 in GSE18520 database; (b) differentially expressed gene analysis was performed under the threshold of ∣logFC > 1∣ and *P* value < 0.05 in GSE27651 database; (c) differentially expressed gene analysis was performed under the threshold of ∣logFC > 1∣ and *P* value < 0.05 in GSE54388 database; (d) five genes were commonly upregulated in GSE18520, GSE27651, and GSE54388 databases, which were also risk factors; (e) six genes were commonly downregulated in GSE18520, GSE27651, and GSE54388 databases, which were also protective factors.

**Figure 3:** PDP1 was overexpressed in ovarian cancer tissue. Notes: (a): the expression pattern of PDP1 in pan-cancer; (b–e): PDP1 was overexpressed in ovarian cancer tissue compared with the normal tissue in TCGA+GTEx, GSE18520, GSE27651, and GSE54388 databases; (f, g): the representative immunohistochemistry image of PDP1 in ovarian cancer and normal tissue.

**Figure 4:** Clinical and prognosis correlation of PDP1 in ovarian cancer. Notes: (a) the expression level of PDP1 in patients with or without lymphatic invasion; (b) the expression level of PDP1 in patients with or without venous invasion; (c) the expression level of PDP1 in stage II/III and stage IV patients; (d–f) the prognosis difference between PDP1 low and high ovarian cancer patients (OS, DSS, and PFI); (g–i) the prognosis prediction efficiency of PDP1 in OS, DSS, and PFI; (j) univariate analysis of PDP1; (k) multivariate analysis of PDP1.

**Figure 5:** PDP1 promotes cell proliferation, invasion, and migration of ovarian cancer. Notes: (a) the expression level of PDP1 in ovarian cancer cell lines; (b, c) the knockdown efficiency of PDP1 in A2780 and SKOV3 cell lines; (d, e) CCk8 assay was performed to evaluate the cell proliferation ability; (f) Transwell assay was performed to evaluate the invasion and migration ability of cancer cells.

**Figure 6:** Biological enrichment of PDP1. Notes: (a) GSEA analysis of PDP1 based on Hallmark gene set; (b) GO analysis of PDP1; (c) KEGG analysis of PDP1.

**Figure 7:** Immune infiltration and drug sensitivity analysis. Notes: (a) CIBERSORT algorithm was performed to explore association between PDP1 and immune cell infiltration; (b–e) the association between PDP1 and drug chemosensitivity.

## Data Availability

The datasets used and/or analysed during the current study are available from the corresponding author on reasonable request.

## Abbreviations

OC: Ovarian cancer
TCGA: The Cancer Genome Atlas
GEO: Gene Expression Omnibus
GSEA: Gene Set Enrichment Analysis
PDP1: Pyruvate dehydrogenase phosphatase catalytic subunit 1
PDKs: Pyruvate dehydrogenase kinases
PDPs: Pyruvate dehydrogenase phosphatases.
